RETRACTED

# Syndecan-1 suppresses cell growth and migration via blocking JAK1/STAT3 and Ras/Raf/MEK/ERK pathways in human colorectal carcinoma cells

**DOI:** 10.1186/s12885-019-6381-y

**Published:** 2019-11-29

**Authors:** Shaojun Wang, Xiaofei Zhang, Guimei Wang, Bin Cao, Hong Yang, Lipeng Jin, Mingjuan Cui, Yongjun Mao

**Affiliations:** 1 Department of Gastroenterology, The Affiliated Hospital of Qingdao University, Qingdao, 266000 China; 2 Department of Geriatrics, The Affiliated Hospital of Qingdao University, No.59 Haier Road, Laoshan District, Qingdao, 266000 Shandong China; 3 Emergency Department, The Affiliated Hospital of Qingdao University, Qingdao, 266000 China

**Keywords:** Syndecan-1, Colorectal carcinoma, Migration, JAK1/STAT3, Ras/Raf/MEK/ERK

## Abstract

**Background:**

Syndecan-1 (SDC-1) is a crucial membrane proteoglycan, which is confirmed to participate in several tumor cell biological processes. However, the biological significance of SDC-1 in colorectal carcinoma is not yet clear. An objective of this study was to investigate the role of SDC-1 in colorectal carcinoma cells.

**Methods:**

Expression of SDC-1 in colorectal carcinoma tissues was evaluated by Reverse transcription-quantitative real-time PCR (RT-qPCR) and western blot. After transfection with pcDNA3.1 or pc-SDC-1, the transfection efficiency was measured. Next, SW480, SW620 and LOVO cell viability, apoptosis, migration and adhesion were assessed to explore the effects of exogenous overexpressed SDC-1 on colorectal carcinoma. In addition, the influences of aberrant expressed SDC-1 in Janus kinase 1 (JAK1)/signal transducer and activator of transcription 3 (STAT3) and rat sarcoma virus (Ras)/rapidly accelerated fibrosarcoma (Raf)/mitogen-activated protein kinase (MEK)/extracellular signal-regulated kinase (ERK) pathways were detected by western blot analysis.

**Results:**

SDC-1 mRNA and protein levels were down-regulated in human colorectal carcinoma tissues. SDC-1 overexpression inhibited cell proliferation via suppressing CyclinD1 and c-Myc expression, meanwhile stimulated cell apoptosis via increasing the expression levels of B-cell lymphoma-2-associated x (Bax) and Cleaved-Caspase-3. Additionally, SDC-1 overexpression restrained cell migration via inhibiting the protein expression of matrix metallopeptidase 9 (MMP-9), and elicited cell adhesion through increasing intercellular cell adhesion molecule-1 (ICAM-1). Furthermore, SDC-1 overexpression suppressed JAK1/STAT3 and Ras/Raf/MEK/ERK-related protein levels.

**Conclusions:**

In general, the evidence from this study suggested that SDC-1 suppressed cell growth, migration through blocking JAK1/STAT3 and Ras/Raf/MEK/ERK pathways in human colorectal carcinoma cells.

RETRACTED

## Background

Colorectal carcinoma is one of the most common malignancies of alimentary canal, which arises from the colon or the junction of the rectum and sigmoid colon. Colorectal carcinoma is generally unrecognized with symptomless in the early stage or is seen with ordinary symptoms in cancer metaphase, such as bloating and indigestion. With growing new cases being diagnosed all around the world every year, colorectal carcinoma is known to be one of the most critical popular diseases, accompanying by a high malignant degree and mortality [1]. Surgical operation and chemotherapy have been developed for the treatment of colorectal carcinoma [2, 3]. Nevertheless, there has been no satisfactory change in the patients survival rate, especially for colorectal carcinoma patients with cancer metastasis which was the dominating cause for poor survival and prognosis of patients [4]. Thus, it is urgent to explore novel targets that may provide potential resolutions for metastasis in colorectal carcinoma cells.

Heparan sulfate proteoglycan (HSPG) is a kind of heparan sulfate (HS)-bonding glycoproteins [5]. Syndecan-1 (SDC-1), the most crucial membrane proteoglycan, is implicated in several cellular processes, such as cell-extracellular matrix interactions [6], growth factor [7], integrin activity [8], migration [9] and inflammatory response [10]. Furthermore, there is growing evidence that SDC-1 participates in the development of tumor progression. For instance, recent evidence suggested that silencing SDC-1 led to cell apoptosis of human urothelial carcinoma [11]. SDC-1 was believed to modulate the cancer stem cell phenotype via regulating inflammatory cytokines in breast cancer [12]. Beyond that, SDC-1 functioned in epithelial-mesenchymal transition and migratory ability in human oral carcinomatosis [13]. A clinic pathological study showed that epithelial SDC-1-positive was significantly associated with tumor size in human colorectal carcinoma [14]. Immunohistochemical research such as that conducted by Yosuke et al. shown that there was unambiguous relativity between loss of SDC-1 and poor prognosis of colorectal carcinoma patients [15]. However, there is no data on the possible role of SDC-1 in human colorectal carcinoma.

In this paper, we verified the mRNA and protein expression of SDC-1 in human colorectal carcinoma tissues and focused on the biological cellular effects of SDC-1 on human colorectal carcinoma cell lines (SW620, SW480 and LOVO), by evaluating cell viability, apoptosis, migration and adhesion. Furthermore, the involved potential signaling pathways were also studied. This study might provide a meaningful opportunity to advance our knowledge of the mechanism of SDC-1 in human colorectal carcinoma, highlighting new therapeutic strategy for the colorectal carcinoma treatment.

RETRACTED

## Methods

### Clinical specimens

A total of 20 patients with colorectal carcinoma were investigated. Between February 2018 to February 2019, 20 patients with colorectal carcinoma were submitted to surgery with resection of colorectal carcinoma in the Affiliated Hospital of Qingdao University (Qingdao, China). Before surgery, no patients have accepted any radiation or chemotherapy. The twenty pairs of tissues were obtained from colorectal carcinoma and from the corresponding peritumor mucosa. For clinical research, the proceeding authorization from each patient and ethical confirmation from the Medical Ethics Committee of the Affiliated Hospital of Qingdao University were obtained.

### Cell culture

Human colorectal cancer cell lines SW620 (CCL-227) and SW480 (CCL-228) were obtained from American Type Culture Collection (ATCC, Manassas, VA, USA) and were cultivated in Leibovitz’s L-15 Medium (ATCC) contained 10% fetal bovine serum (FBS, Gibco). LOVO cells (TCHu 82) were purchased from the Shanghai Cell Bank (Chinese Academy of Sciences, Shanghai, China) and were cultivated in dulbecco’s modified eagle medium (DMEM, Gibco) which was rich in 10% FBS. All cells were placed in a humidified incubator balanced with 5% CO_2_ at 37 °C. All cell lines were authenticated by short tandem repeats (STR) profiling (done by Cobioer, Nanjing, China). None of the cells were contaminated with mycoplasma.

### Cell transfection

The integrated length of SDC-1 was inserted into the control vector (pcDNA3.1, Thermo Fisher, Waltham, MA, USA). The recombination vector was named as pc-SDC-1. The lipofectamine 2000 reagent (Life Technology, Carlsbad, CA, USA) was employed for cell transfection. After 48 h, transfected cells were harvested with the highest transfection efficiency.

### Reverse transcription-quantitative real-time PCR (RT-qPCR)

Trizol reagent (Solarbio, Beijing, China) was used to isolate total RNA from tissue samples or cell cultures. cDNA was synthesized from total RNA by utilizing SuperRT cDNA Synthesis Kit (Cwbio, Jiangsu, China). SYBR® Green PCR Kit (Qiagen, Hilden, Germany) was used for qPCR analysis to detect SDC-1 expression. qPCR was executed on iQ5 Real-Time PCR Detection system (Bio-Rad, Hercules, CA, USA). The mRNA expression of SDC-1 was normalized by β-actin. The relative quantification of SDC-1 in tumor tissues or cells was calculated using 2^-ΔΔCt^ [16, 17].

### Cell viability assay

Cells (5 × 10^3^/well) were seeded in 96-well plates and were cultivated for 48 h. pcDNA3.1 or pc-SDC-1 was transfected to colorectal cancer cells according to the grouping. Then, the Cell Counting kit-8 solutions (CCK-8, Solarbio) were added to each well (10 μL/well). Afterwards, the cell cultures were incubated for 1 h at 37 °C. The OD_450_ was estimated by Microplate Reader (Bio-Rad).

RETRACTED

### Cell apoptosis assay

Cell apoptotic potential was assessed by utilizing propidium iodide (PI)/fluorescein isothiocyanate (FITC)-Annexin V staining kit (Invitrogen, Carlsbad, CA, USA). Specifically, 1 × 10^6^ cells were seeded into 6-well plates and cultured for 48 h. pcDNA3.1 or pc-SDC-1 was transfected to colorectal cancer cells. Then cells were treated with PI (100 μg/mL) and Annexin V-FITC (20 mg/mL) solutions. FACS can (Becton Dickinson San Jose, CA, USA) was used to perform flow cytometry. Finally, FlowJo software (Becton Dickinson) was utilized to calculate the apoptotic cell rate.

### Cell migration assay

Transwell culture chamber (Corning Cosatar, Corning, NY, USA) was utilized for determining the cell migratory ability. The Transwell chamber comprised an 8 μm pore polycarbonate membrane. After transfection, 1 × 10^4^ cells were suspended in 200 μL serum-free medium and seeded into the top chamber. Then 600 μL complete medium was added to the under chamber. After incubation at 37 °C for 24 h, cells that migrated through the membrane were fixed with methanol (Solarbio) and stained with 0.4% crystal violet solutions (Solarbio). Then the numbers of migrated cells were counted under an inverted microscope Inverted Microscope (Olympus).

### Cell adhesion assay

Ten mg/mL fibronectin solutions (500 μL/well) were used to pretreat the 12-well plate for 12 h. The plate was rinsed with phosphate buffer saline (PBS, Solarbio) thrice and then blocked by utilizing 1% bovine serum albumin (BSA, Solarbio) for 1 h. Next, 1 × 10^5^ cells (per well) were transfected with pcDNA3.1 or pc-SDC-1 and cultured for 1 h at 37 °C. Then the suspended solids were removed by PBS. The adhesive cells were fixed with methyl alcohol and dyed with Giemsa stain solution (Solarbio). The numbers of adhesive cells were counted under an Inverted Microscope (Olympus, Shinjuku Monolith, Japan).

### Western blot

Cells were lysed with radio immunoprecipitation assay (RIPA) lysis buffer (Beyotime Biotechnology, Shanghai, China). Super-Bardford Protein Assay Kit (Cwbio) was used to quantify protein concentration. The extracted proteins (10 μL per well) were loaded into 12% polyacrylamide gel on the Bis-Tris Gel system (Bio-Rad) and then transferred to polyvinylidene fluoride (PVDF) membranes. Primary antibodies were prepared in 5% blocking buffer and used to incubate with the membrane at 4 °C overnight. The antibodies included anti-SDC-1 (#ab128936, Abcam, Cambridge, MA, USA), anti-CyclinD1 (#ab16663, Abcam), anti-c-Myc (#ab32072, Abcam), anti-B-cell lymphoma-2-associated x (Bax, #ab77566, Abcam), anti-Cleaved-Caspase-3 (#ab49822, Abcam), anti-matrix metallopeptidase 9 (MMP-9, #ab137867, Abcam), anti-intercellular cell adhesion molecule-1 (ICAM-1, #ab 109,361, Abcam), anti-p-janus kinase 1 (JAK1, #ab138005, Abcam), anti-t-JAK1 (#ab133666, Abcam), anti-p-signal transducer and activator of transcription 3 (STAT3, #ab32143, Abcam), anti-t-STAT3 (#ab137803, Abcam), anti-rat sarcoma virus (Ras, #ab16907, Abcam), anti-rapidly accelerated fibrosarcoma (Raf, #ab230850, Abcam), anti-p-mitogen-activated protein kinase (MEK, #9154, Cell signaling technology, CST, Boston, MA, USA), anti-t-MEK (#9122, CST), anti-p-extracellular signal-regulated kinase (ERK, #9101, CST), anti-t-ERK (#9102, CST) and anti-β-actin (#ab179467, Abcam). Then the membranes were rinsed. The horseradish peroxidase (HRP)-conjugated goat anti-rabbit Immunoglobulin G (IgG, #ab6721, Abcam) were added and incubated with the membranes for 1 h at room temperature. After rinsing, the membranes were treated with the ChemiDoc™ XRS system (Bio-Rad). The chemiluminescence signals were captured and the intensity of the bands was quantified by utilizing Image Lab™ Software (Bio-Rad). Quantification of protein levels was normalized to β-actin.

RETRACTED

### Statistical analysis

Every group of experimentation was repeated 3 times. The results were shown as the mean + standard deviation, which were performed by statistical software of Graphpad 6.0 (San Diego, CA, USA). The *p*-values were calculated by utilizing analysis of variance (ANOVA) and Student's *t*-test. The *p*-value of < 0.05 was considered as a statistically significant result.

## Results

### SDC-1 was down-expressed in human colorectal carcinoma tissues

First of all, we examined SDC-1 expression in human colorectal carcinoma tissues by RT-qPCR. As displayed in Fig. 1a, compared with the corresponding paracancerous tissues, SDC-1 mRNA expression was down-regulated in human colorectal carcinoma specimens (*p* < 0.001). Additionally, three of the twenty tissues were selected for western blot analysis. As shown in Fig. 1b, three colorectal carcinoma tissues exhibited lower expression levels of SDC-1 protein, in comparison with adjacent tissues. These results demonstrated that SDC-1 was down-expressed in human colorectal carcinoma tissues. To further evaluate the effect of SDC-1 expression on cell behaviors in human colorectal carcinoma cells, we constructed pc-SDC-1 plasmid, which contained the full length of SDC-1. pcDNA3.1 or pc-SDC-1 was respectively introduced to SW620 and SW480 cells. The SDC-1 mRNA and protein expression were significantly up-regulated in pc-SDC-1-transfected group, compared with that in pcDNA3.1-transfected group (*p* < 0.001, Fig. 1c-d), hinting efficient overexpression of SDC-1 in human colorectal carcinoma cell lines.

RETRACTED

**Fig. 1:** SDC-1 was down-expressed in human colorectal carcinoma tissues. **a** The mRNA expression of SDC-1 in human colorectal carcinoma tissues (*n* = 20) and the adjacent non-tumor tissues (*n* = 20) was measured by RT-qPCR. **b** The protein expression of SDC-1 in three cases of colorectal carcinoma tissues was determined by western blot. pcDNA3.1 or pc-SDC-1 was transfected into SW620 and SW480 cell lines. Specific overexpression of SDC-1 was confirmed by (**c**) RT-qPCR and (**d**) western blot. β-actin was used as an internal reference for normalizing the expression of SDC-1 protein. ***p < 0.001

### SDC-1 inhibited cell growth of human colorectal carcinoma cells

To explore the functional effect of SDC-1 in human colorectal carcinoma cells, we tested the cell viability and apoptosis of SW620 and SW480 cell lines. Figure 2a presented that overexpressed SDC-1 decreased SW620 and SW480 cell viability (*p* < 0.001). Quite the opposite, it was confirmed by using flow cytometry that the percentage of apoptotic cells was significantly increased in pc-SDC-1 overexpressed group, compared with pcDNA3.1 group (*p* < 0.001, Fig. 2b). Meanwhile, western blot revealed that overexpressed SDC-1 reduced the protein levels of cell-cycle regulators (CyclinD1 and c-Myc), whereas elicited the protein levels of pro-apoptotic factors (Bax and Cleaved-Caspase-3) (*p* < 0.001, Fig. 2c-h). Moreover, the anti-growth effects of overexpressing SDC-1 were presented in LOVO cells. Overexpression of SDC-1 suppressed LOVO cell growth by inhibiting viability and eliciting cell apoptotic ability, which was in accompaniment with the declination of CyclinD1 and c-Myc proteins expression and the enhancement of Bax and Cleaved-Caspase-3 protein levels (*p* < 0.001, Additional file 1: Figure S1). The above-mentioned consequences gave evidence of the inhibitory effect of SDC-1 on cell growth in human colorectal carcinoma cells.

**Fig. 2:** SDC-1 inhibited cell growth of human colorectal carcinoma cells. pcDNA3.1 or pc-SDC-1 was transfected into SW620 and SW480 cell lines. **a** Cell viability was assessed by CCK-8 assay and the absorbance was measured at 450 nm. **b** Flow cytometry analysis to evaluate the percentage of apoptotic cells. **c**-**e** Western blot analysis was utilized to evaluate the expression levels of SDC-1, CyclinD1 and c-Myc. **f**-**h** Western blot analysis was utilized to evaluate the expression levels of SDC-1, Bax and Cleaved-Caspase-3. β-actin was used as an internal reference for normalizing the protein expression. ***p < 0.001

RETRACTED

### SDC-1 suppressed cell migration and promoted cell adhesion of human colorectal carcinoma cells

Subsequently, we assessed the effects of SDC-1 on cell migration and adhesion in SW620 and SW480 cell lines. Transwell assays revealed that SDC-1 attenuated colorectal carcinoma cell migration (*p* < 0.001, Fig. 3a). As displayed in Fig. 3b, the relative adhesion rate were elevated in pc-SDC-1 group, compared with that in pcDNA3.1 group (*p* < 0.001), indicating that SDC-1 overexpression promoted cell adhesion of SW620 and SW480 cell lines. In addition to cell behaviors changes, overexpressed SDC-1 induced the significant decline of pro-metastasis protein expression (MMP-9) and the increase of ICAM-1 protein levels (*p* < 0.001, Fig. 3c-d). Besides, the anti-migratory and pro-adhesion functions of overexpressing SDC-1 were also showed in LOVO cells. Overexpression of SDC-1 attenuated LOVO cell migration by impeding MMP-9 expression and increased cell adhesion by elevating ICAM-1 protein level (*p* < 0.001, Additional file 2: Figure S2). Collectively, these results manifested that SDC-1 suppressed cell migration and promoted cell adhesion of human colorectal carcinoma cells.

**Fig. 3:** SDC-1 suppressed cell migration and promoted cell adhesion of human colorectal carcinoma cells. pcDNA3.1 or pc-SDC-1 was transfected into SW620 and SW480 cell lines. **a** Cells were seeded in transwell chamber. Migrating cells were stained and were counted under a microscope. **b** Substrate fibronectin proteins were coated, and cell adhesion was measured. **c**-**d** Western blot analysis was utilized to evaluate the expression levels of MMP-9 and ICAM-1. β-actin was used as an internal reference for normalizing the protein expression. ***p < 0.001

### SDC-1 inhibited the phosphorylation of JAK1/STAT3 and Ras/Raf/MEK/ERK pathways

The mechanisms underlying SDC-1-induced human colorectal carcinoma cell behavior was confirmed by western blot. The results showed that in both SW620 and SW480 cell lines, the protein levels of p-JAK1, p-STAT3, Ras, Raf, p-MEK and p-ERK were apparently reduced due to overexpressed SDC-1 (*p* < 0.001, Fig. 4 and Fig. 5). Nevertheless, SDC-1 has no significant effect on the protein expression of t-JAK1, t-STAT3, t-MEK and t-ERK. Additionally, overexpression of SDC-1 also hindered JAK1/STAT3 and Ras/Raf/MEK/ERK pathways in LOVO cells (*p* < 0.001, Additional file 3: Figure S3). Altogether, these aforementioned results indicated that SDC-1 blocked JAK1/STAT3 and Ras/Raf/MEK/ERK pathways in human colorectal carcinoma cells.

RETRACTED

**Fig. 4:** SDC-1 inhibited the phosphorylation of JAK1/STAT3 pathway. pcDNA3.1 or pc-SDC-1 was transfected into SW620 and SW480 cell lines. **a**-**b** Western blot analysis was utilized to evaluate the protein levels of p-JAK1, t-JAK1, p-STAT3 and t-STAT3. β-actin was used as an internal reference for normalizing the protein expression. ***p < 0.001

**Fig. 5:** SDC-1 inhibited the phosphorylation of Ras/Raf/MEK/ERK pathway. pcDNA3.1 or pc-SDC-1 was transfected into SW620 and SW480 cell lines. **a**-**b** Western blot analysis was utilized to evaluate the protein levels of Ras, Raf, p-MEK and p-ERK. β-actin was used as an internal reference for normalizing the protein expression. ***p < 0.001

## Discussion

In spite of the current therapy for colorectal carcinoma improving prognosis evaluation, a multitude of patients suffer from the tumor metastasis of colorectal carcinoma [18]. There are some discrepancies of the 5-year survival rate between metastatic colorectal cancer cases and non-metastatic cases yet. There was an epidemiological evidence indicating that one-fifth confirmed cases showed tumor metastasis in human colorectal carcinoma, that generally metastasized to a variety of organs, including liver, lung and bone [19]. Hence, understanding how SDC-1 functions provides promise for novel therapeutic treatment to relieve tumor metastasis of colorectal carcinoma patients. In the present research, our results presented that SDC-1 was down-expressed in human colorectal carcinoma tissues. Moreover, exogenous overexpression of SDC-1 suppressed cell viability and migration, whereas accelerated cell apoptosis and adhesion in SW620 and SW480 cell lines. Finally, we found that overexpression of SDC-1 interrupted JAK1/STAT3 and Ras/Raf/MEK/ERK pathways in human colorectal carcinoma cells.

SDC-1 is a cell-surface molecule characterized by abnormal expressed in tumor tissues. The meta-analysis demonstrated that SDC-1 expression was lower in colorectal carcinoma tissues and was negatively correlated with the malignancy of colorectal carcinoma [20]. Immunohistochemical experiment revealed the decrease or loss of SDC-1 in colorectal adenocarcinomas [21]. Consistently with previous studies, our data disclosed that SDC-1 mRNA and protein expression were both down-regulated in human colorectal carcinoma tissues. The results indicated that SDC-1 might participate in regulating the development of colorectal carcinoma. An interesting research reported that SDC-1 functioned in a wide spectrum of biological processes, such as cancer cell proliferation and apoptosis [22]. Loss of SDC-1 in multiple myeloma cells inhibited cell growth via binding Wnts and R-spondins [23]. In addition, SDC-1 knockdown led to an enhancement of tumor growth in mice model of colorectal carcinoma [24]. Similarly, in this study, we found that overexpressed SDC-1 inhibited cell viability, and elevated cell apoptosis of SW620 and SW480 cells.

RETRACTED

It was known that CyclinD1 was a crucial protein in cell cycle and was abundant in tumor cells [25]. Meta analysis study suggested the incidence of human colorectal carcinoma was linked to CyclinD1 expression. In addition, c-Myc, a kind of oncogene, was reported to express at high level in several cancers, such as breast tumor, ovarian cancer and colorectal cancer [26, 27]. Correlated researches disclosed that c-Myc was closely related to cancer cell viability and apoptosis and was regarded as potential cancer target [28–30]. This study disclosed that overexpression of SDC-1 not only reduced CyclinD1 and c-Myc expression, but also promoted the levels of pro-apoptosis protein (Bax and Cleaved-Caspase-3). These findings further verified that SDC-1 could suppress cell growth of human colorectal carcinoma.

The key role of SDC-1 was demonstrated in intracellular and extracellular matrix adhesion and migration. The results from Péterfia et al. provided empirical evidence of the association of SDC-1 and migration in human fibrosarcoma cells [31]. Recent study on glioma proved that SDC-1 stimulated cell migration of U251 cell line [32]. The migratory capacity of malignant tumor cells, which is a primary intracellular manifestation of tumor metastasis, becomes an absorbing focus in tumor-related research [33, 34]. The regulation of cell migration is an exceedingly intricate process, with multiple proteins involved, such as integrins and extracellular matrix (ECM) [35, 36]. In this research, we observed that the ectopic expression of SDC-1 inhibited SW620 and SW480 cell migration. Along with these biological effects, we also observed the enhancement at cell adhesion of SDC-1-overexpressed SW620 and SW480 cells.

MMP-9 is expressed in several malignant tumors, where MMP-9 exerts critical function in biological regulation [37]. Immunohistochemistry data suggested the great probability of MMP-9 to locate in tumor edge and the contribution of MMP-9 in colorectal cancer cell migration and invasion [38]. ICAM-1 is a well-known transmembrane glycoprotein which is involved in the progression of cell adhesion and signal transduction [39]. Importantly, ICAM-1 expression was positively correlated with infiltration of colorectal tumor [40]. Additionally, methodology article also indicated that detecting ICAM-1 expression was a vital part of standard adhesion assay [41]. According to this, we discovered that overexpressed SDC-1 attenuated MMP-9 and elicited ICAM-1 protein levels. These findings indicated that SDC-1 might exert an anti-metastatic effect on human colorectal carcinoma.

RETRACTED

After stimulation of outside or receiving information from cell matrix, the intracellular signal networks can modify the protein, crack substrate or transfer the protein to specific location in cells through protein-protein interaction to respond to the post-translational modification and ultimately regulate the behaviors of tumor cells [42]. JAK1/STAT3 signaling pathway is affected by several crucial factors, turning on gene transcription thereby participating cancer biological progression [43]. Preceding research reported that JAK1/STAT3 signaling pathway was interrupted by triptolide, consequently suppressing cell proliferation of colorectal carcinoma [44]. Data from Xue et al. identified that JAK1/STAT3 pathway was activated by iron-CDK1 interaction, resulting in an enhancement of cell proliferation in colorectal carcinoma cells [45]. Beyond that, the Ras/Raf/MEK/ERK pathway is also involved in cancer pathogenesis, being regulated by G-protein-coupled receptors (Ras), which activates the downstream factor (Raf) and MEK and ERK, thereby activating gene transcription [46, 47]. Meanwhile, Ras/Raf/MEK/ERK pathway is like a switch for multiple downstream transduction pathways, such as PI3K/AKT/mTOR pathway and Ral GTPase pathway [48]. In colorectal carcinoma, fork-head box D3 (FOXD3) knockdown markedly increased cell growth, cell invasive ability and then activated Ras/Raf/MEK/ERK pathway [49]. Here, we found that SDC-1 overexpression suppressed the phosphorylation of JAK1/STAT3 and Ras/Raf/MEK/ERK-related proteins in human colorectal carcinoma cells. These findings indicated that JAK1/STAT3 and Ras/Raf/MEK/ERK pathways might be involved in regulating the impacts of SDC-1 on cell growth and metastasis in human colorectal carcinoma cells.

## Conclusions

To sum up, this research confirmed that exogenous overexpression of SDC-1 suppressed cell growth, migration via blocking JAK1/STAT3 and Ras/Raf/MEK/ERK pathways. This study would lay the foundation for the research of SDC-1 and quite aid in the early diagnosis and treatment of colorectal carcinoma.

## Supplementary information

**Additional file 1:** **Figure S1.** SDC-1 inhibited cell growth of human colorectal carcinoma cells. pcDNA3.1 or pc-SDC-1 was transfected into LOVO cells. Specific overexpression of SDC-1 was confirmed by (A) RT-qPCR and (B) western blot. (C) Cell viability was assessed by CCK-8 assay, and the absorbance was measured at 450 nm. (D) Flow cytometry analysis to evaluate the percentage of apoptotic cells. (E) Western blot analysis was utilized to evaluate the expression levels of SDC-1, CyclinD1 and c-Myc. (F) Western blot analysis was utilized to evaluate the expression levels of SDC-1, Bax and Cleaved-Caspase-3. β-actin was used as an internal reference for normalizing the protein expression. ***p < 0.001.

RETRACTED

**Additional file 2: Figure S2.** SDC-1 suppressed cell migration and promoted cell adhesion of LOVO cells. pcDNA3.1 or pc-SDC-1 was transfected into LOVO cells. (A) Cells were seeded in transwell chamber. Migrating cells were stained and were counted under a microscope. (B) Substrate fibronectin proteins were coated, and cell adhesion was measured. (C-D) Western blot analysis was utilized to evaluate the expression levels of MMP-9 and ICAM-1. β-actin was used as an internal reference for normalizing the protein expression. ***p < 0.001.

**Additional file 3: Figure S3.** SDC-1 inhibited the phosphorylation of Ras/Raf/MEK/ERK pathway. pcDNA3.1 or pc-SDC-1 was transfected into LOVO cells. (A-B) Western blot analysis was utilized to evaluate the protein levels of Ras, Raf, p-MEK and p-ERK. β-actin was used as an internal reference for normalizing the protein expression. ***p < 0.001.

## Data Availability

The datasets used and/or analyzed during the current study are available from the corresponding author on reasonable request.

## Abbreviations

ANOVA: Analysis of variance
ATCC: The American Type Culture Collection
Bax: B-cell lymphoma-2-associated x
BSA: Bovine serum albumin
CCK-8: Cell counting kit-8
DMEM: Dulbecco’s modified eagle medium
ECM: Extracellular matrix
ERK: Extracellular signal-regulated kinase
FBS: Fetal bovine serum
FITC: Fluorescein isothiocyanate
FOXD3: Fork-head box D3
HRP: Horseradish peroxidase
HS: Heparan sulfate
HSPG: Heparan sulfate proteoglycan
ICAM-1: Intercellular cell adhesion molecule-1
IgG: Immunoglobulin G
JAK1: Janus kinase 1
MEK: Mitogen-activated protein kinase
MMP-9: Matrix metallopeptidase 9
PBS: Phosphate buffer saline
PI: Propidium iodide
PVDF: Polyvinylidene fluoride
Raf: Rapidly accelerated fibrosarcoma
Ras: Rat sarcoma virus
RIPA: Radio immunoprecipitation assay
RT-qPCR: Reverse transcription-quantitative real-time PCR
SDC-1: Syndecan-1
STAT3: Signal transducer and activator of transcription 3
STR: Short tandem repeats
